# Action Recognition Using Action Sequences Optimization and Two-Stream 3D Dilated Neural Network

**DOI:** 10.1155/2022/6608448

**Published:** 2022-06-13

**Authors:** Xin Xiong, Weidong Min, Qing Han, Qi Wang, Cheng Zha

**Affiliations:** ^1^Information Department, First Affiliated Hospital of Nanchang University, Nanchang 330006, China; ^2^Institute of Metaverse, Nanchang University, Nanchang 330031, China; ^3^Jiangxi Key Laboratory of Smart City, Nanchang 330047, China; ^4^School of Mathematics and Computer Science, Nanchang University, Nanchang 330031, China; ^5^School of Software, Nanchang University, Nanchang 330047, China

## Abstract

Effective extraction and representation of action information are critical in action recognition. The majority of existing methods fail to recognize actions accurately because of interference of background changes when the proportion of high-activity action areas is not reinforced and by using RGB flow alone or combined with optical flow. A novel recognition method using action sequences optimization and two-stream fusion network with different modalities is proposed to solve these problems. The method is based on shot segmentation and dynamic weighted sampling, and it reconstructs the video by reinforcing the proportion of high-activity action areas, eliminating redundant intervals, and extracting long-range temporal information. A two-stream 3D dilated neural network that integrates features of RGB and human skeleton information is also proposed. The human skeleton information strengthens the deep representation of humans for robust processing, alleviating the interference of background changes, and the dilated CNN enlarges the receptive field of feature extraction. Compared with existing approaches, the proposed method achieves superior or comparable classification accuracies on benchmark datasets UCF101 and HMDB51.

## 1. Introduction

Action recognition [1–3] has received wide attention from academic communities due to its wide applications in areas, such as behaviour analysis and public safety in smart city. Internet of Things devices collect surveillance videos in the city and analyze the data by using an artificial intelligence system with the fusion of edge and cloud computing. Action recognition is an important application in a smart city. As a result of the interference of complex background in industrial scenarios, the recognition accuracy of this method is low, which is why it is rarely effectively used in practice. The proposed method is committed to improving and solving the problem of the poor effect of action recognition by reducing interferences and extracting discriminative action feature in practical application. An action has two crucial and complementary feature cues, namely, appearances and temporal information [4, 5]. The appearances contain spatial information of action and scene information. The temporal information connects action spatial information from video frames to construct an action line. Assessing the effectiveness of an action recognition system or algorithm can be measured by how well spatial and temporal features are extracted to some extent. These spatial and temporal information provide discriminative action features. References [1–5] focused on spatial and temporal feature extraction and representation. However, extracting feature information is difficult due to many challenges, such as scene changes, different viewpoints, and camera movements. Hence, designing an effective and robust action recognition algorithm and system is crucial. In recent years, deep learning [6] has progressed considerably in image-based object and scene classification [7–10] and recognition [11–14]. It has also been successfully used in human action recognition. However, deep learning in video has failed to achieve the same level of progress as deep learning in image and many problems have yet to be solved.

The action recognition problem is primarily a classification issue. Existing methods have two outstanding problems. First, most existing methods cannot accurately recognize actions because of the interference of background changes caused by not reinforcing the proportion of high-activity action areas and by using the RGB flow only or in combination with the optical flow. Second, the accuracy of some methods that extract action features from RGB video only is influenced by changes in background, angle, illumination, and other factors. Other methods use optical flow as the supplementary modality and not only extract the action feature but also mix the change information of background. The optical flow fails to extract and represent the structure feature of the human body. The skeleton flow is introduced, which can fully represent the feature information of human motion without the interference of scene changes, to focus on action recognition. The RGB flow contains more interference. Our approach does not simply discard RGB information but also fuses the features of two modalities. The motivation of the proposed method is to strengthen high-activity action portions by optimized sampling and by combining the skeleton and RGB information for discriminative feature extraction. Existing works do not focus on improvement of these two parts. Thus, a method using action sequences optimization and two-stream 3D dilated neural network with different modalities for action recognition is proposed in this paper. This method reconstructs the video by reinforcing the proportion of high-activity action areas. A two-stream 3D dilated neural network is then constructed to integrate the features of RGB and skeleton modalities. The academic contributions of this study are as follows:

1. The action sequences optimization method based on shot segmentation and dynamic weighted sampling reconstructs the video by reinforcing the proportion of high-activity action areas, eliminating redundant interval, and extracting long-range temporal information.
2. A two-stream 3D dilated convolution neural network integrates features of RGB and human skeleton information is also proposed. The human skeleton information strengthens the deep representation of humans for robust processing and alleviates the interference of background changes, and the dilated convolution neural network (CNN) enlarges the receptive field of feature extraction.

The rest of this paper is organized as follows. A review of existing studies is presented in Section 2. The proposed method is described in Sections 3to 5. Experimental and evolution results are discussed in Section 6. The conclusion is drawn in Section 7.

## 2. Related Works

Many studies on action recognition have focused on datasets [15, 16] and action classification [17–20] in recent years. Action recognition is difficult to achieve due to large intraclass otherness, nondeterminacy of different actions, and difficult-to-annotate large-scale datasets. Many researchers have focused on action recognition using convolution networks [21–24] and applications [7–9]. Action recognition and object detection have similar notions in technology. Object recognition and action representation are achieved using statistical models of local video descriptors. Unlike object detection, actions are characterized using spatiotemporal evolution of motion with appearance. Descriptors, such as histograms of optical flow and histograms of oriented gradient [25], have been successfully used for action recognition in practice. These methods can only be effective for feature analysis and recognition of a few actions under many constraints. Visual representations learned from CNNs [26] have demonstrated more advantages than hand-crafted features from static images [27–29]. Consistent with previous results of studies that use hand-crafted features, motion-based CNNs perform better than single RGB inputs [30]. Several recent works have proposed CNN extensions for action recognition in video. Some methods utilize deep architectures with 2D-CNN to extract invariance features from some video sequences and achieve satisfactory results even when modality fusion and temporal modelling with sparse sampling for eliminating redundant information are ignored [8–10]. However, these methods are insufficient for big datasets with many classifications. The 3D-CNN provides a simple and effective strategy for extending 2D convolutions to process videos, address the problem, and encode spatial and temporal features simultaneously. Although 3D-CNNs [24, 31] can demonstrate satisfactory performance, these approaches learn video representations for RGB input only and extract temporal features from some continuous frames. Finite video frames can only aggregate short-term temporal features, lacking long-range temporal extraction ability. Moreover, the large number of parameters from each 3D convolution filter increases the computational burden. Reference [1] incorporated two CNNs to fuse motion and appearance features, as well as learning appearance and temporal feature from raw RGB flow frames and optical flow, respectively. Reference [32] adapted methods for action recognition in videos with simple average pooling and multiscale temporal window integration. These methods experiment with multiple modalities that complement lacking features as input. The methods that use optical flow as the supplementary modality not only extract the action feature but also mix the background change information, resulting in low accuracy.

The long short-term memory- (LSTM-) based approach [33] uses a spatial-temporal dual-attention network to extract the high-level semantics features from fully connected layers and spatial features from middle-level convolution layers. In [34], a structured adaptive video summarization method was proposed, which integrates shot segmentation and video summarization into a hierarchical structure-adaptive recurrent neural network. To reward the summary generator under the assistance of the video reconstructor, Zhao et al. [35] proposed a dual learning framework to capture both the spatial and temporal information of the summary and provide more guidance for the summary generator. Although these methods have a strong ability to extract temporal features, they have a weak ability to extract action spatial features. The attention-based method [36] proposed a spatiotemporal attention network to learn the discriminative feature representation for actions by respectively characterizing the beneficial information at the frame level and the channel level. Zhao et al. [37] proposed a coattention model-based recurrent neural network (CAM-RNN) for video processing, where the CAM is utilized to encode the visual and text features and the RNN works as the decoder to generate the video caption. These methods do not perform well enough for long temporal feature extraction.

Some methods based on a multistream structure have made new achievements. References [38–40] constructed multistream networks to extract action features, thus greatly improving the recognition accuracy and providing inspiration for related work. Reference [38] proposed a novel human-related region-based multistream convolution neural network for action recognition. The improved block-sparse robust principle component analysis is proposed to avoid noise. Reference [39] proposed an ActionS-ST-VLAD approach to aggregate video spatiotemporal features for action recognition with the consideration of encoding deep features both in subactions spatially and in action stages temporally. Reference [40] first proposed a spatiotemporal saliency-based video object segmentation model to extract an actor and its most motion salient body part. Then, a two-stream network (TS-Net) is designed to extract semantics features. These three heuristic methods use optical flow as recognition modality, which contains more interferential background information, thus reducing the accuracy. Garcia et al. [41] proposed a distilled multistream method and designed an interstream connection mechanism to improve the learning process of the hallucination work. Reference [42] proposed a two-stream method by introducing LSTM in spatial flow and DenseNet in temporal flow to extract spatial and temporal action features. These two methods ignore the noise interference and extract long-range features by enlarging the receptive field and eliminating redundant frames.

In the graph-based method [43], a two-stream graph convolution network (GCN) was proposed to adaptively extract features from the coordinates of joints. A multistream GCN based on hidden conditional random field model is proposed in [44] to boost the performance by retaining the spatial structure of human joints from beginning to end. Only when the structural modelling of human body is accurate can these methods achieve good accuracy. However, the oversmoothing issue constrains the accuracy. These methods do not focus on increasing the proportion of high-activity action areas, eliminating redundant intervals, and extracting long-range temporal information.

Most existing methods cannot accurately recognize actions because of the interference of background changes caused by not reinforcing the proportion of high-activity action areas and by using the RGB flow only or in combination with the optical flow. The interference of background in RGB flow or optical flow changes influences the accuracy. To alleviate these problems, an action recognition method that uses action sequences optimization and two-stream fusion network with different modalities is proposed. The action sequences optimization method is based on shot segmentation and dynamic weighted sampling. It reconstructs the video by reinforcing the proportion of high-activity action areas, eliminating redundant intervals, and extracting long-range temporal information. A two-stream 3D dilated CNN that integrates the features of RGB and human skeleton information is proposed as well. The human skeleton information strengthens the deep representation of humans for robust processing and alleviates the interference of background changes, and the dilated CNN enlarges the receptive field of feature extraction.

## 3. Overview of the Proposed Method

Accurate extraction of action features is important. The proposed two-stream 3D dilated neural network for action recognition is illustrated in this section.  Figure 1 shows the two components of the proposed method for action recognition. The first component is the action sequences optimization module. The input video is divided into several video cubes in accordance with the shot segmentation algorithm [45]. The video is then reconstructed using the proposed dynamic weighted algorithm to optimize and recreate action sequences. The optimized action sequences module refines the video to increase the ratio of action features. Then, the reconstructed video flows to the second component, the two-stream 3D dilated neural network module. A two-stream CNN is constructed to extract features of two supplementary modalities, namely, RGB and human skeleton, to strengthen the deep representation of humans for robust processing and enlarge the receptive field of feature extraction. The network fuses the advantages of two modalities. Class score fusion then yields the final prediction.

## 4. Action Sequences Optimization Method

The majority of existing methods process video sequences averagely to extract action features without reinforcing the proportion of high-activity action areas. Even though some methods are aware of it, they do not process the relationship between the high-activity and low-activity action areas properly. Redundant frame parts typically found in video datasets are a challenge in action recognition. The noise interference from redundant frame parts in a video negatively influences the computational cost and performance of the method and reduces the ability and efficiency of the algorithm to focus on the action. We attempt to solve these issues in this section. The action sequences optimization method is based on shot segmentation and dynamic weighted sampling. It reconstructs the video by reinforcing the proportion of high-activity action areas, eliminating redundant intervals, and extracting long-range temporal information.

### 4.1. Shot Segmentation

Videos generally have many scenes or shot cuts and redundant sequence parts, which are a challenge in action recognition. The noise interference from redundant parts in the video has an unpredictable influence on action recognition and reduces the ability and efficiency of the algorithm to focus on the action. Videos are a sequence of frames. The change of scene or shot cut causes interference in action feature extraction. A reasonable video segmentation method for shot cut is crucial. Our research dataset HMDB51 contains many videos with two or three shot cuts. Effective action information is typically found in only one shot. Hence, shot segmentation in video is an important research topic.

An existing method such as that presented in [32] segments the video sequences into fixed three parts on average and not according to the shot changes, which may destroy the underlying hierarchical structure of the video. It is a process of video sequence segmentation, not shot segmentation. Therefore, the action feature is averagely processed in the network. The method we used for segmenting the video is according to the shot cut changes to detect the video shot boundary and preserve the underlying hierarchical structure of the video, as referred to in a previous study [45]. The method based on key frames or semantic information does not consider the problem of shot boundary switching, thus causing the video sequence to contain more interference information. The proposed method extracts more features by processing the sequences that contain more action information. The proposed method applies a structural analysis process to detect shot boundaries; this process consists of two steps: (1) candidate shot segment selection and (2) cut transition detection. Each frame in the video should be represented mathematically. To reduce the computational overhead and make execution faster, only the blue plane, which is most sensitive plane and contains maximum information, is used instead of the three RGB planes for extracting features. The visual feature is extracted using pixel-wise distance [46] between frames and then it is used to extract potential candidate segments. Segments are then optimized and detected using the cut transition detection algorithm based on discrete cosine transform or horizontal and vertical coefficients [45]. A vector is formed by systematically choosing 10 values from the cosine transform of each frame, and the cosine distance between these vectors is used for cut transition detection.

Then, we utilize the dynamic weighted sampling algorithm, which reinforces the proportion of high-activity action areas and allows the sequence to contain more action features for recognition.

### 4.2. Dynamic Weighted Sampling Algorithm

After video shot segmentation, a dynamic weighted sampling algorithm is used to reconstruct the optimized action video. The redundant parts are filtered by focusing on dynamic weighted sampling. A single video is typically divided into one to three shot parts given the characteristics of datasets. We then reference the method in [47] to compare the entropy of different shot parts. The video shot with maximum entropy contains nearly complete action information. Thus, we design an algorithm for dynamic sampling of different shots with varying entropy weights, average sampling, or random sampling, as shown in Figure 2.

One frame is sampled in a shot of every *T* frame in average sampling. We set *T*_average_=2 in this study. One shot is divided uniformly as a part for every *T* frame, and one frame is randomly sampled from each part in random sampling. If one shot is excessively short, then the algorithm pads the shot with the last frame to the length of *T* or *nT* frames. In this study, we set *T*_random_=4. The sampling rate is 1/*T*. Finally, segments are reconstructed to an optimized video after sampling.

The single video in datasets can be divided into a maximum of three shot parts by using the shot segmentation algorithm. This condition presents the following situations: Situation1={Seg_1_}, Situation2={Seg_1_,  Seg_2_}, and Situation3={Seg_1_,  Seg_2_, Seg_3_}, where Seg_ _ is the segment. In Situation1, we set the average sampling rate to 1/2 to obtain optimum results.  Table 1 shows the performance comparison of different sampling rates in various datasets. The accuracy of Situation1 and the original video is nearly the same but the workload and computation are reduced by half.

In Situation2, the algorithm compares the entropy of Seg_1_ and Seg_2_, and the frequency of segment with larger entropy is set to 1/2 in average sampling. Random sampling is also performed in another set. As shown in Table 2, Seg_1_ <  Seg_2_. Four possibilities are experimented and, with the factor that reduces the computational burden taken into account, the proposed setup is the best choice.

In Situation3, the algorithm compares the entropy of Seg_1_, Seg_2_, and  Seg_3_, with the assumption that  Seg_2_ has the largest entropy segment. The sampling rate of the segment with the largest entropy is set to 1/2 and others are set to 1/4 with random sampling. Four sampling rate possibilities are tested, and their accuracies are compared in Table 3.

Algorithm 1 describes the proposed action sequences optimization algorithm. The input is RGB video sequences, and the output is reconstructed video sequences. First, the input video is divided into three segments by using the shot cut method. Second, the video segments are ranked according to entropy information. Third, sampling weights are assigned dynamically, and the videos are reconstructed into an optimized video. The average sampling rate is 1/2, and the random sampling rate is 1/4. The action sequences optimization method processes the time dimension of videos without additional labels. After one video is sampled into a relatively short length, 3D-CNN is used to optimize the video sequence after the reconstruction.

## 5. Two-Stream 3D Dilated Neural Network

The extraction of action features of several existing methods from RGB videos alone influences the accuracy via changes in background, angle, illumination, and other factors. Other methods use the optical flow as the supplementary modality and not only extract the action feature but also mix the change information of the background. How to strengthen and extract the action feature from original RGB data is a challenge.  Figure 3 shows the RGB, optical flow, and skeleton flow frames of an action. The proposed neural network uses multiple modalities, skeleton frame sequences, and RGB sequences, which is used to deal with these issues and strengthens the deep representation of humans for robust processing. Different networks and modalities have varying specialties for extracting and representing various features. Appropriate modalities can be used to extract useful features accurately. The RGB flow contains both useful information and useless information. Given the unexplainable nature of CNNs, identifying an action from the scene is possible. For example, the horse area in video frames may be the key point to action recognition in the ride-horse subset in HMDB51 and the green land space dominates most of the video frames of the soccer penalty subset in UCF101. Extracting background features has both advantages and disadvantages. The neural network may have difficulty generalizing effective action characteristics of the same action in different scenes when the extracted scene feature information is greater than the action feature information. This scenario is equivalent to sacrificing the ability of the network to focus on the motion itself while constantly trying to fit the characteristic information of scenes. The skeleton flow is introduced, which can fully represent the feature information of human motion without the interference of scene changes, to focus on action recognition. However, skeleton information alone is insufficient in classifying similar actions, such as eating and drinking, talking and chewing, and flic-flac and handstand. Only actions with small intraclass and large interclass differences can easily be recognized accurately when skeleton feature information is extracted. The advantage of action recognition in skeleton features is the absence of background information interference that allows the neural network to focus on the action itself. Intuitively discarding information, especially contextual information, can degrade the performance. However, the proposed method only removes background information in skeleton flow and still retains complete video information in RGB flow. Our approach does not simply discard information but fuses the features of two modalities.

Thus, a two-stream CNN that integrates features of RGB and human skeleton information is also proposed in this study. The human skeleton information strengthens the deep representation of humans for robust processing and alleviates the interference of background changes, and the dilated CNN enlarges the receptive field of feature extraction to achieve superior or comparable performance. The original RGB data combined with processed skeleton data make the feature extraction more accurate. Unlike 2D convolution, 3D convolution extracts both temporal and spatial features from multiple sequences simultaneously. Temporal information is ignored in the 2D convolution, which extracts features from the local neighborhood on feature maps with an applied bias. The result is then subjected to activation. A unit value at position (*a*, *b*) in the feature map is expressed in formula (1):

(1) $$\begin{array}{c} {\text{Value}}^{ab}=\text{relu}\left(t\overset{H-1}{\underset{h=0}{\sum }}\overset{W-1}{\underset{w=0}{\sum }}xy^{\left(a+h\right)\left(b+w\right)}+z\right), \end{array}$$

where relu(*∗*) represents the rectified linear activation function; *t* and *x* are iterable parameters in the feature map; *H* and *W* are the height and width parameters, respectively; and *z* is the bias. The 2D-CNN is applied to extract spatial features only. The video data issue must capture the action feature in consecutive frames. The 3D convolutions extract both spatial and temporal features. At each feature map of any single layer, the value at position (*a*, *b*, *c*) in the feature map is expressed in formula (2):

(2) $$\begin{array}{c} {\text{Value}}^{abc}=\text{relu}\left(t\overset{H-1}{\underset{h=0}{\sum }}\overset{W-1}{\underset{w=0}{\sum }}\overset{D-1}{\underset{d=0}{\sum }}xy^{\left(a+h\right)\left(b+w\right)\left(c+d\right)}+z\right), \end{array}$$

where *d* is the 3D kernel size of the temporal dimension; relu(*∗*) is the rectified linear activation function; *t* and *x* are iterable parameters; *H* and *W* are the height and width parameters, respectively; and *z* is the bias. Hence, the 3D convolution kernel with a size of 3 × 3 × 3 is utilized to construct our two-stream 3D dilated neural network. Satisfactory results are obtained from modelling the temporal information using 3D convolution and pooling layers. On the basis of 3D-CNN, we introduce dilated processing into the proposed network.  Figure 4 illustrates the 3D dilated convolution operation.

On the basis of the original convolution kernel, the dilated convolution enlarges the receptive field by inserting rows and columns with weight of 0 between features. In this paper, the parameter of dilation rate *r* is used to represent the number of inserted rows and columns. Therefore, formula (3) is transformed into the following formula (3):

(3) $$\begin{array}{c} {\text{Value}}^{abc}=\text{relu}\left(t\overset{H-r}{\underset{h=0}{\sum }}\overset{W-r}{\underset{w=0}{\sum }}\overset{D-r}{\underset{d=0}{\sum }}xy^{\left(a+h\right)\left(b+w\right)\left(c+d\right)}+z\right). \end{array}$$

*r*=2 means that the 3D kernel size increased from 3 × 3 × 3 to 5 × 5 × 5. The architecture of the two-stream 3D dilated convolution network is constructed for both flows with 7 convolution layers, 5 max-pooling layers, and 1 fully connected and softmax layer with a stride of 1. The sizes of the first two and the last three pooling kernels are 1 × 2 × 2 and 2 × 2 × 2, respectively, as shown in Figure 5. The input of skeleton flow is obtained from the pose estimation algorithm [48]. A deep or stacked network is unnecessary for extracting action features because of the absence of interference in the background and the action sequences optimization method. Finally, each flow obtains the corresponding class scores before the classification we referred to in [53] to fuse the scores of the two networks. Scores of the two streams are fused to predict the action label.

## 6. Experiments

### 6.1. Implementation Setup and Datasets

Experiments are implemented on a workstation equipped with 3.3 GHz Intel(R) Xeon(R) E-2 CPU, 24 GB RAM, NVIDIA RTX A5000 GPU, and Linux Ubuntu 18.04. The preprocessing procedure consists of two steps. First, the input video is optimized to reconstruct the video sequences. Second, the pose estimation algorithm processes the video into skeleton data. The proposed deep learning method is applied via PyTorch. The shot cut method is referenced in [45] and the pose estimation algorithm is referenced in literature [48]. The proposed algorithm is implemented in MATLAB 2019a using OpenCV3.2.0 with CUDA. The two-stream 3D dilated network with RGB and skeleton modalities has the following network parameters for training: batch size and momentum of 32 and 0.9, respectively; 60,000 maximum iterations; and initial learning rate of 0.001, which decreases to 1/10 every 15,000 iterations. In the validation procedure, the batch size is set to 32, and the mirror is set to false.

The experiments are conducted on two challenging action datasets, namely, UCF101 and HMDB51. These two datasets contain trimmed video data, so the videos reconstructed by action sequences optimization are labeled according to the classification of the original dataset. The action sequences optimization method processes the time dimension of videos without additional labels. The UCF101 [15] dataset, a widely used benchmark for action recognition, contains approximately 13,000 clips from YouTube. Each video lasts an average of 7 seconds. A total of 2.4 million frames are distributed among 101 different action categories, including five kinds of movements, namely, human and object interaction, body movement, interpersonal interaction, playing musical equipment, and various kinds of sports. Specific examples are applying eye makeup, baby crawling, handstand walk, soccer penalty kick, and volleyball spiking. Videos have a resolution and frame rate of 320 × 320 pixels and 25 fps, respectively. The HMDB51 dataset [16] consists of nearly 7,000 videos with 51 kinds of actions. The majority of videos are from movies, with some from public databases and online video libraries, such as Google and YouTube. Each category contains at least 101 samples, such as laughing, kissing, firing a gun, waving, and riding a bike. The resolution and frame rate of these videos are 320 × 240 pixels and 30 fps, respectively.

### 6.2. Ablation Study

A novel action recognition method that uses action sequences optimization and two-stream 3D dilated network with different modalities is proposed. The action sequences optimization method based on shot segmentation and dynamic weighted sampling reconstructs the video by reinforcing the proportion of high-activity action areas, eliminating redundant intervals, and extracting long-range temporal information. A two-stream 3D dilated CNN that integrates the features of RGB and human skeleton information is also proposed. The human skeleton information strengthens the human information, thus alleviating the interference of background changes, and the dilated CNN enlarges the receptive field of feature extraction.

#### 6.2.1. Evaluation of Action Sequences Optimization Method

The use of action sequences optimization is an important innovation in action recognition. Most existing methods cannot accurately recognize actions because of the interference of background changes caused by not reinforcing the proportion of high-activity action areas. The action sequences optimization method is based on shot segmentation and dynamic weighted sampling. It reconstructs the video by reinforcing the proportion of high-activity action areas, eliminating redundant intervals, and extracting long-range temporal information. We compare the accuracy of the original and reconstructed action video using the action sequences optimization method. The results prove the superiority of the proposed method. Experiment results on the two datasets are presented in Table 4. We also analyze the computational cost. The running time for training of the proposed method is presented in Table 5.

#### 6.2.2. Evaluation of Two-Stream 3D Dilated Neural Network

Some methods extract action features from RGB videos only, where the accuracy is influenced by changes in background, angle, illumination, and other factors. Other methods use optical flow as the supplementary modality. They not only extract the action feature but also mix the change information of the background, thereby causing weak attention to the target and missing important features from different modalities. The proposed two-stream CNN that integrates the features of RGB and human skeleton information overcomes the challenges of inaccurate extraction of action features in RGB. The human skeleton information strengthens the deep representation of human action, thus alleviating the interference of background changes, and the dilated CNN enlarges the receptive field of feature extraction. Experiments are conducted on UCF101 and HMDB51 datasets to prove the effectiveness and superiority of the proposed method. Experimental data in Table 6 indicate that the single RGB flow or skeleton flow performs worse than the fusion network. The accuracy of RGB flow is interfered by the background, and the skeleton flow is influenced by the feature representation of large intraclass gaps and small interclass gap, thus achieving relatively low accuracy. The proposed method fuses these two complementary modalities, and the experiment demonstrates the effectiveness of the two-stream 3D dilated neural network with two modalities.

### 6.3. Comparison with State-of-the-Art Methods

In this section, the proposed method is compared with state-of-the-art action recognition approaches. The performance of the method based on feature engineering to extract action features and classification is far inferior to that of the proposed method, which lacks action semantic features [49, 50]. As a result of the interference of background, the method based on traditional TS-Net does not accurately extract the action features and ignores the extraction of skeleton features, which causes the method to be less robust and accurate [31, 42, 51–57]. The methods in [38, 40, 46, 54, 58–78] are interfered by redundant parts and ignore the attention of action features. Thus, the extra part will negatively affect the accuracy of action feature extraction. The proposed method is compared with state-of-the-art methods, and the results are shown in Table 7. The training time taken to learn the model for UCF101 and HMDB51 is 4.5 and 3.5 hours, respectively. Benchmark datasets are used to validate the robustness of the proposed method, which achieves superior or comparable classification accuracies. The trends and merits of the model are given as follows:

1. The action sequences optimization method reconstructs the video. It reinforces the proportion of high-activity action areas, eliminates redundant intervals, and extracts long-range temporal information.
2. The two-stream 3D dilated neural network integrates features of RGB and human skeleton information. It strengthens feature representation with robustness and alleviates the interference of background changes. The dilated CNN enlarges the receptive field of feature extraction.

In general, our proposed method recognizes actions successfully in most cases. In some cases, the skeleton information is insufficient in classifying similar actions, such as eating and drinking, as well as talking and chewing, thus decreasing the accuracy of using RGB only. To classify similar actions, we plan to fuse the GCN to further extract coordinate features in the future. To verify the performance of the proposed method on the large-scale action recognition dataset, experiments on the Kinetics dataset [80] were conducted. As shown in Table 8, the proposed method achieves comparable classification accuracy. Compared with these approaches, the proposed method eliminates redundant intervals and enlarges the receptive field by introducing dilated convolution with different modality to extract long-range and discriminative feature.

Experiments were conducted on different networks to test the flexibility of the proposed method.  Table 9 shows the proposed method compared with the traditional single-stream 3D network that fuses RGB and skeleton modalities. The method with modality fusion performs better, and the results show the effectiveness of the proposed method.

## 7. Conclusion

A novel action recognition method using action sequences optimization and two-stream 3D dilated neural network with different modalities is proposed in this study. The action sequences optimization method based on shot segmentation and dynamic weighted sampling reconstructs the video by reinforcing the proportion of high-activity action areas, eliminating redundant intervals, and extracting long-range temporal information. A two-stream 3D dilated neural network that integrates features of RGB and human skeleton information is proposed. The human skeleton information strengthens the human deep representation for robust processing and alleviates the interference of background changes, and the dilated CNN enlarges the receptive field of feature extraction. The proposed method achieves superior or comparable classification accuracies on two challenging datasets. The application of the proposed method could enhance the intelligence ability of video surveillance systems in smart cities and improve the accuracy of existing action recognition methods. Further research will improve hierarchical action feature extraction on large datasets through the attention mechanism and aggregate more features through transformer encoding longer sequences.

## Figures and Tables

**Figure 1:** Overview of the proposed method. The optimized action sequences module reconstructs the input video to increase the ratio of action features. The network fuses the advantages of two modalities and enlarges the receptive field of action feature.

**Figure 2:** Dynamic weighted sampling. In one shot, the different sampling strategy can obtain different reconstructed videos of reconstruct.

**Figure 3:** Comparisons of different modalities. The RGB and optical flow mix the change information of the background and the action information. The skeleton flow contains the human action information only, which strengthens the deep representation of humans for robust processing.

**Figure 4:** 3D dilated convolution operation.

**Figure 5:** Structure of the two-stream 3D dilated network.

**Algorithm 1:** Proposed action sequences optimization algorithm.

**Table 1:** Accuracy comparison of different sampling rates of Situation1 (%).

Sampling rate	UCF101	HMDB51
1/8	69.65	51.13
1/4	89.29	66.88
1/2	93.93	72.05
1	69.65	51.13

**Table 2:** Accuracy comparison of different sampling rates of Situation2 (%).

Sampling rate (Seg_1_, Seg_2_)	UCF101	HMDB51
1/8, 1/2	92.13	70.79
1/4, 1/2	95.17	75.36
1/2, 1/2	89.45	68.52
1, 1/2	92.99	72.86

**Table 3:** Accuracy comparison of different sampling rates of Situation3 (%).

Sampling rate (Seg_1_, Seg_2_, Seg_3_)	UCF101	HMDB51
1/4, 1/2, 1/8	93.84	73.88
1/4, 1/2, 1/4	95.85	75.93
1/4, 1/2, 1/2	92.60	69.27
1/4, 1/2, 1	92.38	68.57

**Table 4:** Accuracy evaluation of the action sequences optimization method (%).

	UCF101	HMDB51
The original video	91.13	66.48
Reconstructed action video	**95.56**	**75.26**

**Table 5:** Comparison of the running time for training of the proposed method (hours).

	UCF101	HMDB51
The original video	20.5	18
Reconstructed action video	**17.5**	**16**

**Table 6:** Evaluation of performance of different modalities (%).

	UCF101	HMDB51
RGB flow + 3D dilated only	89.15	66.09
Skeleton flow + 3D dilated only	68.84	43.62
Two-stream fusion network	**95.56**	**75.26**

**Table 7:** Accuracy comparison of different methods (%).

	UCF101	HMDB51
Peng et al. [49]	87.9	61.1
Zhao et al. [35]	89.1	65.1
Tran et al. [31]	85.3	62.3
Tu et al. [38]	94.5	69.8
Tu et al. [40]	94.8	70.4
Zhao et al. [42]	92.5	—
Wang et al. [79]	92.4	62.0
Feichtenhofer et al. [51]	92.5	65.4
Qiu et al. [52]	93.7	66.3
Wang et al. [53]	92.4	70.5
Lu et al. [54]	90.4	65.0
Hara et al. [55]	90.7	63.8
Cong et al. [56]	91.8	68.8
Wang et al. [58]	84.0	55.1
Sun et al. [59]	91.9	70.0
Huang et al. [60]	92.6	69.1
Yao et al. [60]	92.1	65.9
Liu et al. [62]	92.5	62.4
Hao et al. [63]	93.7	66.7
Tong et al. [64]	94.6	69.4
Li et al. [65]	91.5	63.0
Peng et al. [66]	94.0	68.7
Long et al. [67]	94.6	69.2
Wang et al. [68]	94.9	70.2
Wu et al. [69]	94.3	70.9
Li et al. [70]	94.5	70.2
Cai and Hu [71]	91.0	64.7
Cai and Hu [71]	92.5	66.5
Li et al. [73]	86.7	—
Xu et al. [74]	**96.3**	**76.3**
Jiang et al. [75]	94.6	70.7
Yang and Zou [76]	92.7	—
Chang et al. [77]	93.8	—
Deng et al. [78]	95.3	71.3
Wang et al. [57]	94.5	74.1
Proposed method	95.6	75.3

**Table 8:** The accuracy comparison of different methods on Kinetics dataset (%).

	Top-1	Top-5
Tran et al. [31]	56.1	79.5
Feichtenhofer et al. [51]	56.0	77.3
Donahue et al. [80]	57.0	79.0
Wang et al. [32]	69.1	83.7
Zolfaghari et al. [81]	68.0	80.9
Jiang et al. [82]	73.1	90.6
Proposed method	69.6	87.1

**Table 9:** Accuracy comparison of different network (%).

	UCF101	HMDB51
Tran et al. [31]	85.3	62.3
Tran et al. [31] + modality fusion	90.2	68.5
Proposed method	95.6	75.3

## Data Availability

All data used in this paper can be obtained by contacting the authors of this study.
